# Review on Diagnosis of COVID-19 from Chest CT Images Using Artificial Intelligence

**DOI:** 10.1155/2020/9756518

**Published:** 2020-09-26

**Authors:** Ilker Ozsahin, Boran Sekeroglu, Musa Sani Musa, Mubarak Taiwo Mustapha, Dilber Uzun Ozsahin

**Affiliations:** ^1^Department of Biomedical Engineering, Near East University, Nicosia / TRNC, Mersin-10, 99138, Turkey; ^2^DESAM Institute, Near East University, Nicosia / TRNC, Mersin-10, 99138, Turkey; ^3^Department of Artificial Intelligence Engineering, Near East University, Nicosia / TRNC, Mersin-10, 99138, Turkey

## Abstract

The COVID-19 diagnostic approach is mainly divided into two broad categories, a laboratory-based and chest radiography approach. The last few months have witnessed a rapid increase in the number of studies use artificial intelligence (AI) techniques to diagnose COVID-19 with chest computed tomography (CT). In this study, we review the diagnosis of COVID-19 by using chest CT toward AI. We searched ArXiv, MedRxiv, and Google Scholar using the terms “deep learning”, “neural networks”, “COVID-19”, and “chest CT”. At the time of writing (August 24, 2020), there have been nearly 100 studies and 30 studies among them were selected for this review. We categorized the studies based on the classification tasks: COVID-19/normal, COVID-19/non-COVID-19, COVID-19/non-COVID-19 pneumonia, and severity. The sensitivity, specificity, precision, accuracy, area under the curve, and F1 score results were reported as high as 100%, 100%, 99.62, 99.87%, 100%, and 99.5%, respectively. However, the presented results should be carefully compared due to the different degrees of difficulty of different classification tasks.

## 1. Introduction

Coronaviruses have been around for many decades, and it has affected many animals/mammal species and human being. By March 11, 2020, the World Health Organization (WHO) [1] declared the new coronavirus called the COVID-19, a pandemic, and it has brought the entire globe into a compulsory lockdown. Coronavirus is a family of RNA viruses that is capable of causing significant viral pathogens in humans and animals. Corona is medium-sized viruses with the largest viral RNA genome known. Coronavirus infects both birds and mammals, but the bat is host to the largest number of the viral genotype of coronavirus. So, the bat is the host and does not get infected. It can, however, spread the virus to a human. As of 24^th^ of August 2020, there have been more than 23 million confirmed cases of coronavirus worldwide, with about 800,000 of such cases resulting in the death of the infected patient. This is spread around 216 countries, areas, or territories. However, around five million infected patients have recovered worldwide [2]. The USA, Brazil, India, and Russia are the top four countries with the highest number of cases. Around 90 million tests have conducted in China, followed by the USA, Russia, and India, with 72 million, 33 million, and 32 million tests, respectively [2].

Testing COVID-19 involves analyzing samples that indicate the present or past presence of severe acute respiratory syndrome-associated coronavirus 2 (SARS-CoV-2). The test is done to detect either the presence of the virus or of antibodies produced in response to infection. COVID-19 diagnostic approach is mainly divided into two broad categories, a laboratory-based approach, which includes point of care-testing, nucleic acid testing, antigens tests, and serology (antibody) tests. The other approach is using medical imaging diagnostic tools such as X-ray and computed tomography (CT) [3].

The laboratory-based tests are performed on samples obtained via nasopharyngeal swab, throat swabs, sputum, and deep airway material [4]. The most common diagnostic approach is the nasopharyngeal swab, which involves exposing a swab to paper strips containing artificial antibodies designed to bind to coronavirus antigens. Antigens bind to the strips and give a visual readout [4]. The process is pretty fast and is employed at the point of care. The nucleic acid test has low sensitivity between 60-71% [4]. On the other hand, Fang et al. [5] showed that radiologic methods could provide higher sensitivity than that of lab tests.

The use of medical imaging tools is the second approach of COVID-19 virus detection. These tools are playing an important role in the management of patients that are confirmed or suspected to be infected with the virus. It is worthy of note that without clinical suspicion, findings from X-ray, or CT images are nonspecific as many other diseases could have a similar pattern [6].

Thoracic CT scan is the imaging modality of choice that plays a vital role in the management of COVID-19. Thoracic CT has a high sensitivity for diagnosis of COVID-19 which makes it a primary tool for COVID-19 detection [5]. CT scan involves transmitting X-rays through the patient's chest, which are then detected by radiation detectors and reconstructed into high-resolution medical images. There are certain patterns to look out for in a chest CT scans which present themselves in different characteristic manifestations. The potential findings with 100% confidence for COVID-19 in thoracic CT images are ground − glass opacity (GGO) ± crazy − paving and consolidation, air bronchograms, reverse halo, and perilobular pattern [6].

The abovementioned findings are reports presented by a radiologist who specializes in interpreting medical images. Interpretation of these findings by expert radiologists does not have a very high sensitivity [4]. Artificial intelligence (AI) has been employed as it plays a key role in every aspect of COVID-19 crisis management. AI has proven to be useful in medical applications since its inception, and it became widely accepted due to its high prediction and accuracy rates. In the diagnosis stage of COVID-19, AI can be used to recognize patterns on medical images taken by CT. Other applications of AI include, but not limited to, virus detection, diagnosis and prediction, prevention, response, recovery, and to accelerate research [7]. AI can be used to segment regions of interest and capture fine structures in chest CT images, self-learned features can easily be extracted for diagnosis and other applications as well. A recent study showed that AI accurately detected COVID-19 and was also able to differentiate it from other lung diseases and community-acquired pneumonia [8]. In this study, we review the diagnosis of COVID-19 by using chest CT toward AI.

## 2. Materials and Methods

We searched ArXiv, MedRxiv, and Google Scholar for AI for COVID-19 diagnosis with chest CT. At the time of writing (August 24, 2020), there have been nearly 100 studies and only 17 of them were peer-reviewed papers. In total, 30 studies (17 peer-reviewed and 13 non-peer-reviewed papers) were selected for this review. We noticed that very different classification terms are reported by the authors such as “normal”, “healthy”, “other”, “COVID-19”, “non-COVID-19”, “without COVID-19”, “community-acquired pneumonia (CAP)”, “other pneumonia”, “bacterial pneumonia”, “SARS”, “lung cancer”, “type A influenza (influ-A)”, and “severity”. Therefore, we categorized the studies into four main tasks as follows: COVID-19/normal, COVID-19/non-COVID-19, COVID-19/non-COVID-19 pneumonia, and COVID-19 severity classification. COVID-19 group consists of COVID-19 patients. The normal group includes only healthy subjects. Non-COVID-19 group includes either one of the cases which is not COVID-19 or a combination of all other cases. The non-COVID-19 pneumonia group includes other types of pneumonia, which is not caused by COVID-19, such as viral or bacterial pneumonia, as well as influenza A and SARS. Lastly, COVID-19 severity classification aims at classifying the COVID-19 cases as severe or nonsevere.

Since the rapid studies on the detection of COVID-19 in CT scans continue, the researchers who take into account the peer-review period in the journals share the results they obtained in their studies with other researchers and scientists as preprints in different publication environments. Machine learning is used to make decisions on tasks that people have difficulty making decisions or problems that require more stable decisions using both numerical and image-based data. A deep convolutional neural network (CNN) is the most widely used among machine learning methods. It is one of the first preferred neural networks, especially in image-based problems, since it contains both feature extraction and classification stages and produces very effective results. In image-based COVID-19 researches, the CNN model or different models produced from CNN are widely encountered. In the researches, a generally hold-out method and a few *k*-fold cross-validation were used during the training phase. In the hold-out method, while training is done by dividing the data into two parts as test and train, in *k*-fold cross-validation, the data is divided into *k*-folds, and the folds are trained *k*-times by shifting the testing fold in each training so that each fold is used in the test phase. It is used as a better method for model evaluation.

## 3. Results

### 3.1. COVID-19/Normal Classification Studies

Alom et al. [9] implemented two deep learning models for COVID-19 detection and segmentation. Inception Recurrent Residual Neural Network (IRRCNN), which is based on transfer learning, was used for the COVID-19 detection task, and the NABLA-N model was for the segmentation task. They considered different datasets to detect COVID-19 on CT images, by using an additional chest X-ray dataset. The publicly available dataset was considered for the segmentation procedure of CT images, and the dataset that consists of 425 CT image samples, with 178 pneumonia, and 247 normal images were considered for the COVID-19 detection purpose. All images were resized to the dimensions of 192 × 192 pixels, and 375 of total images were used for training and validation with a data augmentation procedure. The training was performed using Adam optimizer with a learning rate of 1 × 10^−3^ and a batch size of 16. The COVID-19 detection and segmentation accuracy were achieved by 98.78% and 99.56%, respectively.

Hu et al. [10] constructed an AI model on ShuffleNet V2 [11], which provides fast and accurate training in transfer learning applications. The considered CT dataset consists of 521 COVID-19 infected images, 397 healthy images, 76 bacterial pneumonia images, and 48 SARS images. The data augmentation procedure as flip, rotation, translation, brightness adjustment, and flip+brightness adjustment was applied in this study to increase the number of training images. The first experiment was performed on the classification of COVID-19 images from normal healthy images. The average sensitivity, specificity, and area under the curve (AUC) score were obtained as 90.52%, 91.58%, and 0.9689, respectively.

Gozes et al. [12] proposed a comprehensive system to detect COVID-19 from normal cases. The proposed system included lung segmentation, COVID-19 detection in CT slices, and marking case as COVID-19 using a predetermined threshold based on the counted COVID-19 positive slices. Several datasets were considered in training and testing phases, and pretrained network ResNet50 was used for the detection of COVID-19. The sensitivity, specificity, and the AUC score were achieved as 94%, 98%, and 0.9940, respectively.

In another study for differentiation of COVID-19 from normal cases, Kassani et al. [13] used several pretrained networks such as MobileNet [14], DenseNet [15], Xception [16], InceptionV3 [17], InceptionResNetV2 [18], and ResNet [19] to extract the features of images within the publicly available dataset. Then, extracted features were trained using six machine learning algorithms, namely, decision tree, random forest, XGBoost, AdaBoost, Bagging, and LightGBM. Kassani et al. [13] concluded that the Bagging classifier obtained the optimal results with a maximum of 99.00% ± 0.09 accuracy on features extracted by pretrained network DesnseNet121.

Jaiswal et al. [20] implemented a pretrained network DenseNet201-based deep model on classifying 2,492 CT-scans (1,262 positive for COVID-19, and the rest 1,230 are negative) as positive or negative. They compared their results with VGG16, ResNet152V2, and Inception-ResNetV2. They concluded that their model outperformed other considered models and achieved an overall accuracy of 96.25%.  Table 1 summarizes the studies on COVID-19 vs. normal cases.

### 3.2. COVID-19/Non-COVID-19 Classification Studies

Jin et al. [30] considered 496 COVID-19 positive and 260 negative images collected in Wuhan Union Hospital, Western Campus of Wuhan Union Hospital, and Jianghan Mobile Cabin Hospital in Wuhan. Besides, they used two publicly available international databases, LIDC-IDRI [28] and ILD-HUG [31] (1012 and 113 subjects, respectively) as negative cases to develop the system. A 2D convolutional neural network was used for the segmentation of CT slices, and then, a model was trained for positive and negative cases. Jin et al. reported that the proposed system achieved the AUC score of 0.9791, sensitivity of 94.06%, and specificity of 95.47% for the external text cohort.

Singh et al. [32] proposed a multiobjective differential evolution- (MODE-) based convolutional neural networks to detect COVID-19 in chest CT images. It was concluded that the proposed method outperformed the CNN, ANFIS, and ANN models in all considered metrics between 1.6827% and 2.0928%.

Amyar et al. [33] developed another model architecture that included image segmentation, reconstruction, and classification tasks, which was based on the encoder and convolutional layer. The experiments were performed on three datasets that included 1044 CT images, and the obtained results showed that the proposed architecture achieved the highest results in their experiment, with 0.93% of the AUC score.

Ahuja et al. [34] used data augmentation and pretrained networks to classify COVID-19 images. Data augmentation was performed using stationary wavelets, and the random rotation, translation, and shear operations were applied to the CT scan images. ResNet18, ResNet50, ResNet101, and SqueezeNet were implemented for the classification task, and Ahuja et al. concluded that ResNet18 outperformed other models by obtaining a 0.9965 AUC score.

Liu et al. [35] proposed another deep neural network model, namely, lesion-attention deep neural networks, where the backbone of the model used the weights of pretrained networks such as VGG16, ResNet18, and ResNet50. The proposed model was capable of classifying COVID-19 images, which was the main aim of the study, with 0.94 of the AUC score using VGG16 as the backbone model. Besides this, the model was able to make a multilabel prediction on the five lesions.

Instead of deep learning approaches, Barstugan et al. [36] considered machine learning algorithms to classify 150 COVID-19 and non-COVID-19 images. Several feature extraction methods such as grey-level size zone matrix (GLSZM) and discrete wavelet transform (DWT) were considered in the feature extraction process, and the extracted features were classified using a support vector machine. *K*-fold cross-validations were performed in the experiments with 2, 5, and 10 folds. Barstugan et al. concluded that 99.68% of accuracy was achieved by SVM using the GLSZM feature extraction method.

Wang et al. [37] conducted another study on differentiating COVID-19 from non-COVID-19 CT scans. In their proposed network, UNet was first trained for lung region segmentation, and then, they used a pretrained UNet to test CT volumes to obtain all lung masks. They concatenated CT volumes with corresponding lung masks and sent them to the proposed DeCoVNet for the training. Wang et al. concluded that the proposed network achieved a 0.959 ROC AUC score.

Chen et al. [38] performed a study on collected 46,096 images from 106 patients (Renmin Hospital of Wuhan University–Wuhan, Hubei province, China). The proposed system was based on segmenting CT scans using UNet++ and predicting the COVID-19 lesions. The prediction was performed by dividing an image into four segments and counting the consecutive images. If three consecutive images were classified as containing lesions, the case was classified as positive for COVID-19. The proposed system was evaluated using five different metrics, and it achieved 92.59% and 98.85% of accuracy in prospective and retrospective testing, respectively.

Jin et al. [39] considered the segmentation and pretrained models to classify COVID-19, healthy images, and inflammatory and neoplastic pulmonary diseases. Initially, preprocessing was applied to CT scan images to standardize images that were collected from five hospitals in China. Several segmentation models such as V-Net and 3D U-Net++ were considered, and segmented images were trained using pretrained network ResNet50 [19], Inception networks [17], DPN-92 [40], and Attention ResNet-50 [41]. Jin et al. concluded that the ResNet50 achieved the highest classification rates by 0.9910 of AUC score, 97.40% of sensitivity, and 92.22% of specificity with the images segmented by 3D U-Net++ segmentation model.

Pathak et al. [42] proposed a system for the detection of COVID-19 in CT scans that considered a preproposed transfer learning. The system used the ResNet50 to extract the features from CT images, and a 2D convolutional neural network was considered for the classification. The proposed system was tested on 413 COVID-19 and 439 non-COVID-19 images with 10-fold cross-validation, and it achieved 93.01% of accuracy.

Polsinelli et al. [43] proposed a light architecture by modifying the CNN. The proposed model was tested on two different datasets, and several experiments with different combinations were performed. The proposed CNN achieved 83.00% of accuracy and 0.8333 of F1 score.

Han et al. [44] proposed a patient-level attention-based deep 3D multiple instance learning (AD3D-MIL) that learns Bernoulli distributions of the labels obtained by a pooling approach. They used a total of 460 chest CT examples, 230 CT examples from 79 COVID-19 confirmed patients, 100 CT examples from 100 patients with pneumonia, and 130 CT examples from 130 people without pneumonia. Their proposed model achieved an accuracy, AUC, and the Cohen kappa score of 97.9%, 99.0%, and 95.7%, respectively, in the classification of COVID-19 and non-COVID-19.

Harmon et al. [45] considered 2724 CT scans from 2617 patients in their study. Lung regions were segmented by using 3d anisotropic hybrid network architecture (AH-Net), and the classification of segmented 3D lung regions was performed by using pretrained model DenseNet121. The proposed algorithm achieved an accuracy, specificity, and AUC score of 0.908, 0.930, and 0.949, respectively.  Table 2 shows the summary of the COVID-19/non-COVID-19 classification results.

### 3.3. COVID-19/Non-COVID-19 Pneumonia Classification Studies

Xu et al. [52] proposed a method that consisted of preprocessing, CT image segmentation using ResNet18, and the classification of CT scans performed by adding location-attention that provides the relative location information of the patch on the pulmonary image. The proposed method tested on the considered 618 CT samples (219 with COVID-19, 224 CT images with influenza-A viral, and 175 CT images for healthy people), and Xu et al. concluded that the overall accuracy rate of the proposed method was 86.7%.

Wang et al. [53] proposed another deep learning method to distinguish COVID-19 and other pneumonia types. The segmentation, suppression of irrelevant area, and COVID-19 analysis were the processes of the proposed method. DenseNet121-FPN [15] was implemented for lung segmentation, and COVID19Net that had a DenseNet-like structure was proposed for classification purposes. Two validation sets were considered, and the authors reported 0.87 and 0.88 ROC AUC scores for these validation sets.

In addition to classify COVID-19 and normal cases, Hu et al. [10] performed another experiment to differentiate COVID-19 cases from other cases as bacterial pneumonia and SARS. The average sensitivity, specificity, and the AUC score were obtained as 0.8571, 84.88%, and 92.22%, respectively.

Bai et al. [54] implemented the deep learning architecture EfficientNet B4 [55] to classify COVID-19 and pneumonia slices of CT scans. The diagnosis of the six radiologists on the corresponding patients were used to evaluate the efficiency of the results obtained by an AI model. The AI model achieved 96% of accuracy, while the average accuracy of the diagnosis of radiologists was obtained at 85%.

Kang et al. [56] proposed a pipeline and multiview representation learning technique for COVID-19 classification using different types of features extracted from CT images. They used 2522 CT images (1495 are from COVID-19 patients, and 1027 are from community-acquired pneumonia) for the classification purpose. The comparison was performed using the benchmark machine learning models, namely, support vector machine, logistic regression, Gaussian-naive-Bayes classifier, *K*-nearest-neighbors, and neural networks. The proposed method outperformed the considered ML models with 95.5%, 96.6%, and 93.2% in terms of accuracy, sensitivity, and specificity, respectively.

Another study was performed by Shi et al. [57] to classify COVID-19 and pneumonia. They considered 1658 and 1027 confirmed COVID-19 and CAP cases. Shi et al. proposed a model that is based on random forest and automatically extracted a series of features as volume, infected lesion number, histogram distribution, and surface area from CT images. The proposed method and considered machine learning models (logistic regression, support vector machine, and neural network) were then trained by the selected features with 5-fold cross-validation. The authors reported that the proposed method outperformed other models and produced the optimal AUC score (0.942).

Ying et al. [58] designed a network named as DRE-Net, which is based on the modifications on pretrained ResNet-50. The CT scans of 88 COVID-19 confirmed patients, 101 patients infected with bacteria pneumonia, and 86 healthy persons. The designed network was compared by the pretrained models, ResNet, DenseNet, and VGG16. The presented results showed that the designed network outperformed other models by achieving 0.92 and 0.95 of AUC scores for the image and human levels.

In addition to COVID-19/non-COVID-19 classification, Han et al. [44] performed experiments to classify COVID-19, common pneumonia, and no pneumonia cases as three classes classification. Their proposed AD3D-MIL model achieved an accuracy, AUC, and the Cohen kappa score of 94.3%, 98.8%, and 91.1%, respectively.

Ko et al. [59] proposed a model, a fast-track COVID-19 classification network (FCONet) that used VGG16, ResNet-50, InceptionV3, and Xception as a backbone to classify images as COVID-19, other pneumonia, or nonpneumonia. They considered 1194 COVID-19, 264 low-quality COVID-19 (only for testing), and 2239 pneumonia, normal, and other disease CT scans in their study. All images were converted into grayscale image format with dimensions of 256 × 256. They used rotation and zoom data augmentation procedures to maximize the number of training samples. It was concluded that FCONet based on ResNet-50 outperformed other pretrained models and achieved 96.97% of accuracy in the external validation data set of COVID-19 pneumonia images.

Li et al. [8] proposed a COVNet that used ResNet50 as a backbone to differentiate COVID-19, nonpneumonia, and community-acquired pneumonia. In their study, 4352 chest CT scans from 3322 patients were considered. A max-pooling operation was applied to the features obtained from COVNet using the slices of the CT series, and the resultant feature map was fed to a fully connected layer. This led to generate a probability score for each considered class. It was concluded that the proposed model achieved a sensitivity, specificity, and ROC AUC scores of 90%, 96%, and 0.96, respectively, for the COVID-19 class.

Ni et al. [60] considered a total of 19,291 CT scans from 14,435 individuals for their proposed model to detect COVID-19 in CT scans. Their proposed model included the combination of Multi-View Point Regression Networks (MVPNet), 3D UNet, and 3D UNet-based network for lesion detection, lesion segmentation, and lobe segmentation, respectively. Their algorithm analyzed the volume of abnormalities and the distance between lesion and pleura to diagnose the COVID-19, and it was concluded that the proposed algorithm outperformed three radiologists in terms of accuracy and sensitivity by achieving 94% and 100%, respectively.  Table 3 summarizes the classification results for COVID-19/non-COVID-19 pneumonia cases.

### 3.4. COVID-19 Severity Classification Studies

Xiao et al. [61] implemented a pretrained network ResNet34 to diagnose COVID-19 severity. The experiments were performed using five-fold cross-validation, and 23,812 CT images of 408 patients were considered. They concluded that the model achieved the ROC AUC score of 0.987, and the prediction quality of detecting severity and nonseverity of 87.50% and 78.46%.

Zhu et al. [62] proposed a model that was optimized by traditional CNN and VGG16 to stage the COVID-19 severity. A publicly available dataset was considered, and 113 COVID-19 confirmed cases were used to test their hypothesis. Obtained scores were compared by scores given by radiologists, and it was concluded that the top model achieved a correlation coefficient (*R*^2^) and mean absolute error of 0.90 and 8.5%, respectively.

Pu et al. [63] proposed an approach that initially segmented lung boundary and major vessels at two *t* points using UNet and registered these two images using a bidirectional elastic registration algorithm. Then, the average density of the middle of the lungs was used to compute a threshold to detect regions associated with pneumonia. Finally, the radiologist used to rate heat map accuracy in representing progression. In their study, two datasets that consisted of 192 CT scans were considered.  Table 4 summarizes the key findings of the severity quantification studies.

## 4. Discussion

The 13 of the 30 published articles considered in this review have been published as preprints, while the 17 of them have been published in journals after the peer-review process. Regardless of its form of publication, machine learning and deep learning have been the focus of these studies. In particular, deep learning approaches such as CNN, which performed the feature extraction process automatically, were widely used in these researches.

Besides, pretrained networks were commonly used for the segmentation, feature extraction, and classification stages. Especially DenseNet121, ResNet50, ShuffleNet V2 were successfully reported by the researchers in the classification stages, while successful results were obtained with the images produced by UNet ++ at the segmentation stage. It was pointed out by the researchers that many of the developed systems were modeled using the modifications or improvements pretrained networks to improve the classification accuracy of COVID-19 in CT images after preprocessing and segmentation stages. This has shown that widely used pretrained networks can be used very successfully at every stage of image classification. Some researchers classified COVID-19 cases using machine learning techniques instead of using deep learning approaches by extracting the features from the images and achieved high recognition results. This brings essential advantages in terms of learning speed.

However, while the images used are not standard and performing experiments on different image databases in each research does not make it possible to make a comprehensive comparison, it contributes to deduce general opinion. While the *k*-fold cross-validation is time-consuming, a few of the researches used it, and most of the researchers performed experiments using a hold-out method, which is based on dividing the dataset into training and testing set with defined percentages. However, this makes it challenging to analyze the consistency of the models, but it does not reduce the importance of performed experiments, obtained results, and the role of artificial intelligence in the fight against COVID-19.

## 5. Conclusions

COVID-19 continues to spread around the globe. New classification and prediction models using AI, together with more publicly available datasets, have been arising increasingly. However, the majority of the studies are from the preprint literature and have not peer-reviewed. Furthermore, many of them have different classification tasks. Some of the studies have been conducted with very limited data. The data used in the studies might have come from different institutions and different scanners. Therefore, preprocessing of the data to make the radiographic images more similar and uniform is important in terms of providing more efficient analysis and consistency. The lack of demographic and clinical information of the patients is another limitation of these studies. We believe as the more dataset on COVID-19 with are available, the more accurate studies will be conducted. These findings are promising for AI to be used in the clinic as a supportive system for physicians in the detection of COVID-19.

## Figures and Tables

**Table 1:** COVID-19/normal classification results. Class.: classification; bac. pneu.: bacterial pneumonia; Sens.: sensitivity; Spec.: specificity; Prec.: precision; Acc.: accuracy; AUC: area under the curve; Ref.: reference.

Class.	Subjects	Dataset	Method	Sens. (%) or recall	Spec. (%)	Prec. (%)	Acc. (%)	AUC (%)	F1-score	Ref.
COVID-19/normal	178 pneumonia 247 normal	Private + [21–23]	DL IRRCNN	N/A	N/A	N/A	98.78	N/A	98.85	Alom et al. [9] *Preprint*
COVID-19/normal	521 COVID-19 397 normal 76 bac. pneu. 48 SARS	[24–26]	DL ShuffleNet V2	90.52	91.58	N/A	91.21	96.89	N/A	Hu et al. [10] *Preprint*
COVID-19/normal	106 COVID-19 100 normal	Private + [27, 28]	DL ResNet50	98.2	92.2	N/A	N/A	99.6	N/A	Gozes et al. [12] *Preprint*
COVID-19/normal	COVID-19: X-ray:117; CT:20 normal: X-ray:117; CT:20	[21, 22, 29]	DenseNet121 + Bagging	99.00	N/A	99.00	99.00	N/A	99.00	Kassani et al. [13] *Preprint*
COVID-19/normal	1,262 COVID-19 1,230 normal	[23]	DenseNet201	96.29	96.21	96.29	96.25	97.0	96.29	Jaiswal et al. [20] *Peer-reviewed*

**Table 2:** COVID-19/non-COVID-19 classification results. Class.: classification; Sens.: sensitivity; Spec.: specificity; Prec.: precision; Acc.: accuracy; AUC: area under the curve; Ref.: reference.

Class.	Subjects	Dataset	Method	Sens. (%) or recall	Spec. (%)	Prec. (%)	Acc. (%)	AUC (%)	F1-score	Ref.
COVID-19/ non-COVID-19	496 COVID-19 1385 others	Private + [28, 31]	CNN	94.06	95.47	N/A	94.98	97.91	NA	Jin et al. [30] *Preprint*
COVID-19/ non-COVID-19	N/A	[46]	CNN	~90	~90	N/A	~90	Not clear	~90	Singh et al. [32] *Peer-reviewed*
COVID-19/ non-COVID-19	449 COVID-19 100 normal 98 lung cancer 397 other	Private + [47, 48]	DL multitask	94	79	N/A	86	93	N/A	Amyar et al. [33] *Preprint*
COVID-19/ non-COVID-19	349 COVID-19 397 non-COVID-19	Private + [47, 49]	ResNet18	100.0	98.6	N/A	99.4	99.65	99.5	Ahuja et al. [34] *Peer-reviewed*
COVID-19/ non-COVID-19	564 COVID-19 660 non-COVID-19	[50]	VGG16 based lesion-attention DNN	88.8	N/A	87.9	88.6	94.0	87.9	Liu et al. [35] *Conference proceeding*
COVID-19/ non-COVID-19	53 COVID-19 97 other	Not clear	SVM	97.56	99.68	99.62	98.71	N/A	98.58	Barstugan et al. [36] *Preprint*
COVID-19/ non-COVID-19	313 COVID-19 229 without COVID-19	Private	UNet	90.7	91.1	N/A	90.1	95.9	N/A	Wang et al. [37] *Peer-reviewed*
COVID-19/ non-COVID-19	51 COVID-19 55 control	Private	UNet++	94.34	99.16	N/A	98.85	N/A	N/A	Chen et al. [38] *Preprint*
COVID-19/ non-COVID-19	723 COVID-19 413 others	Private	UNet++ + ResNet-50	97.4	92.2	N/A	N/A	99.1	N/A	Jin et al. [39] *Preprint*
COVID-19/ non-COVID-19	413 COVID-19 439 non-COVID-19	[32, 51]	ResNet-50 + 2D CNN	91.46	94.78	95.19	93.02	N/A	N/A	Pathak et al. [42] *Peer-reviewed*
COVID-19/ non-COVID-19	460 COVID-19 397 non-COVID-19	[26, 47]	CNN SqueezeNet	85.00	81.00	81.73	83.00	N/A	83.33	Polsinelli et al. [43] *Preprint*
COVID-19/ non-COVID	230 COVID-19 130 normal	Private	AD3D-MIL	97.9	NA	97.9	97.9	99.0	97.9	Han et al. [44] *Peer-reviewed*
COVID-19/ non-COVID	1029 COVID-19 1695 non-COVID-19	Private	AH-Net DenseNet121	84.0	93.0	NA	90.8	94.9	NA	Harmon et al. [45] *Peer-reviewed*

**Table 3:** COVID-19/non-COVID-19 pneumonia classification results. Class.: classification; bac. pneu.: bacterial pneumonia; Sens.: sensitivity; Spec.: specificity; Prec.: precision; Acc.: accuracy; AUC: area under the curve; Ref.: reference.

Class.	Subjects	Dataset	Method	Sens. (%) or recall	Spec. (%)	Prec. (%)	Acc. (%)	AUC (%)	F1-score	Ref.
COVID-19/influ-A/normal	219 COVID-19 224 influ-A 175 normal	Private	CNN ResNet	86.7	N/A	81.3	N/A	N/A	83.9	Xu et al. [52] *Peer-reviewed*
COVID-19/CT-EGFR	1266 COVID-19 4106 CT-EGFR	Private	COVID19Net (DenseNet-like str.)	79.35	71.43	N/A	85.00	86.00	90.11	Wang et al. [53] *Peer-reviewed*
COVID-19/other pneu.	521 COVID-19 397 normal 76 bac. pneu. 48 SARS	[26, 47]	DL ShuffleNet V2	85.71	84.88	N/A	85.40	92.22	N/A	Hu et al. [10] *Preprint*
COVID-19/other pneu.	521 COVID-19 665 non-COVID-19 pneu.	Private	DNN EfficientNet B4	95	96	N/A	96	95	N/A	Bai et al. [54] *Peer-reviewed*
COVID-19/CAP	1495 COVID-19 1027 CAP	Private	Multiview representation learning	96.6	93.2	N/A	95.5	NA	N/A	Kang et al. [56] *Peer-reviewed*
COVID-19/CAP	1658 COVID-19 1027 CAP	Private	RF-based ML model	90.7	83.3	N/A	87.9	94.2	N/A	Shi et al. [57] *Preprint*
COVID-19/bac. pneu./normal	88 COVID-19 101 bac. pneu. 86 normal	Private	DRE-Net	96	N/A	79	86	95	87	Ying et al. [58] *Preprint*
COVID-19/other pneu./non-pneu.	230 COVID-19 100 normal	Private	AD3D-MIL	90.5	NA	95.9	94.3	98.8	92.3	Han et al. [44] *Peer-reviewed*
COVID-19/other pneu./non-pneu.	1194 COVID-19 1357 other pneu. 998 normal 444 lung cancer	Private + [26, 47]	FCONet ResNet50	99.58	100.0	NA	99.87	100.0	NA	Ko et al. [59] *Peer-reviewed*
COVID-19/other pneu./non-pneu.	1292 COVID-19 1735 pneumonia 713 non-pneu.	Private	COVNet ResNet50	90	96	NA	NA	96.0	NA	Li et al. [8] *Peer-reviewed*
COVID-19/other pneu./healthy	3854 COVID-19 6871 other pneu. 8566 healthy	Private	MVPNet 3D UNet 3D UNet-based network	100	25	NA	94	NA	97.0	Ni et al. [60] *Peer-reviewed*

**Table 4:** COVID-19 severity classification results. Class.: classification; Sens.: sensitivity; Spec.: specificity; Prec.: precision; AUC: area under the curve; Ref.: reference.

Class.	Subjects	Dataset	Method	Sens. (%) or recall	Spec. (%)	Prec. (%)	AUC (%)	Ref.
COVID-19 severe/nonsevere	23,812 COVID-19	Private	ResNet34	N/A	N/A	81.3	98.7	Xiao et al. [61] *Peer-reviewed*
COVID-19 severity score	131 COVID-19	[21]	CNN VGG16	N/A	N/A	NA	NA	Zhu et al. [62] *Peer-reviewed*
COVID-19 severity and progression	72 COVID-19 120 others	Private	UNet BER Algorithm	95	84	N/A	N/A	Pu et al. [63] *Peer-reviewed*

## Data Availability

The data used to support the findings of this study are included within the article.
